The article "Synthesis and Characterization of a Novel Dual-Responsive Nanogel for Anticancer Drug Delivery" was published in 2022. Journal: Oxid Med Cell Longev.

# Synthesis and Characterization of a Novel Dual-Responsive Nanogel for Anticancer Drug Delivery

**DOI:** 10.1155/2022/1548410

**Published:** 2022-09-19

**Authors:** Darya Aminoleslami, Sahar Porrang, Parviz Vahedi, Soodabeh Davaran

**Affiliations:** ^1^Research Centre for Pharmaceutical Nanotechnology, Tabriz University of Medical Sciences, Tabriz, Iran; ^2^Chemical Engineering Faculty, Sahand University of Technology, Sahand New Town, Tabriz, Iran; ^3^Department of Anatomical Sciences, Maragheh University of Medical Sciences, Maragheh, Iran; ^4^Department of Medical Nanotechnology, Faculty of Advanced Medical Science, Tabriz University of Medical Sciences, Tabriz, Iran

## Abstract

In this study, to reduce the side effects of anticancer drugs and also to increase the efficiency of current drug delivery systems, a pH and temperature-responsive polymeric nanogel was synthesized by copolymerization of N-vinylcaprolactam (VCL) and acrylic acid (AA) monomers (P(VCL-co-AA)) with a novel cross-linker, triethylene glycol dimethacrylate (TEGDMA), as a biocompatible and nontoxic component. The structural and physicochemical features of the P(VCL-co-AA) nanogel were characterized by FT-IR, DLS/Zeta potential, FE-SEM, and ^1^HNMR techniques. The results indicated that spherical polymeric nanogel was successfully synthesized with a 182 nm diameter. The results showed that the polymerization process continues with the opening of the carbon-carbon double bond of monomers, which was approved by C-C band removing located at 1600 cm^−1^. Doxorubicin (Dox) as a chemotherapeutic agent was loaded into the P(VCL-co-AA), whit a significant loading of Dox (83%), and the drug release profile was investigated in the physiological and cancerous site simulated conditions. P(VCL-co-AA) exhibited a pH and temperature-responsive behavior, with an enhanced release rate in the cancerous site condition. The biocompatibility and nontoxicity of P(VCL-co-AA) were approved by MTT assay on the normal human foreskin fibroblasts-2 (HFF-2) cell line. Also, Dox-loaded P(VCL-co-AA) had excellent toxic behavior on the Michigan Cancer Foundation-7 (MCF-7) cell line as model cancerous cells. Moreover, Dox-loaded P(VCL-co-AA) had higher toxicity in comparison with free Dox, which would be a vast advantage in reducing Dox side effects in the clinical cancer treatment applications.

## 1. Introduction

Breast cancer is one of the most widespread cancers among women in the world for many years [1]. Surgery is one of the well-known treatments for breast cancer. By progressing in science, surgery knowledge moved from radical mastectomy to a more conservative form [2]. Although surgical treatment is not recommended for inflammatory breast cancer and recurrent and metastatic forms [2]. However, on the other hand, surgery can cause unresected tumors and increase the rates of local relapse [3]. Therefore, chemotherapy has always been used as the main cancer treatment method. Doxorubicin, as a widely used anticancer, was used to treat numerous varieties of cancers [4]. Most of pharmaceutical agents including doxorubicin have toxic effects on human body [5, 6]. Nanomedicines are becoming very popular these decades for their special properties like small size, reduced drug toxicity, controlled drug release, and ease of biological distribution [7–10]. These properties make nanomedicines be suitable method for personalized treatment in breast cancer management, although up to now no product has been registered. The use of nanomedicines such as nanogels (NGs) as drug nanocarriers is particular for making a balance between maximum therapeutic efficacy and lower toxicity [11–16]. They can control drug release in response to physiological or environmental triggers [15, 17]. NGs are swollen cross-linked polymer nanoparticles that can be used as highly efficient nanocarriers in controlled drug delivery [18]. Biocompatibility, stability, high surface area, easy surface modification, high cellular uptake, and unique mechanical properties are some specific features of NGs, which are important in intracellular delivery applications [19, 20]. Nanogels can be used as smart cancer treatment agents in stimulus-responsive systems category. These systems can control drug release in response to physiological or environmental triggers [12, 21]. Several stimulus-responsive polymers have been utilized for targeted drug delivery. Because of higher metabolism and inflammation [22–24] through tumor tissues, temperature-responsive polymers were introduced for cancer treatment. These polymers are sensitive to ambient temperature changes and classified according to the lower critical solution temperature (LCST). Temperature-responsive polymers are soluble and swollen at temperatures below LCST due to the formation of hydrogen bonds between the hydrophilic portions of the polymer and water molecules. However, at temperatures above LCST, they become insoluble due to the stronger reaction of the hydrophobic groups compared to hydrogen bonds [20, 25–27]. Polymer concentration, solvent auxiliaries, additives, and types of existing functional groups are among the factors affecting the polymer's LCST point. For example, if the hydrophilic groups' counts be higher than hydrophobic groups, due to the augmentation in the possibility of hydrogen bonding between the polymer and water, an increase in LCST temperature can be observed [28, 29]. Poly(N-isopropyl acrylamide) (PNIPAAm) and poly(n-vinylcaprolactam) (PVCL) are among the temperature-sensitive polymers. PNIPAAM is a polymer with a critical solubility point of about 32° C, while its LCST is nonmolecular weight dependent [30]. PVCL is also a polymer with a critical solubility point of about 32-34° C, but its LCST depends on its molecular weight, polymer concentration, and solvent composition [20, 26, 27]. One of the special properties of PVCL is its resistance to amidase enzymes, which naturally produces fewer toxic amides due to the decomposition of the polymer in its environment [19, 31, 32]. Moreover, the pH of cancerous sites is lower than physiological pH due to the high rate of glycolysis in both aerobic and anaerobic conditions. So, pH is one of the factors that can be used in targeted drug delivery [26]. Poly(acrylic acid) (PAA) and poly(methacrylic acid) (PMAA) are some kinds of pH-responsive polymers [33]. PAA responds to the pH of the environment-dependent on the ionization and deionization of the carboxylic group at different pHs [29]. PMAA is another example that changes depending on the separation of its carboxylic acid group [34].

By simultaneously using temperature and pH-responsive monomers in the nanogel structure, dual-responsive systems can be created which have controlled drug release behavior in the cancerous site. Recently, Chang et al. synthesized pH and temperature-responsive nanogels based on sodium alginate with the natural pH sensitivity and PNIPAAm as a temperature-sensitive polymer [35]. They modified sodium alginate by glutamic acid and ethylenediamine to change its charge distribution to achieve desire pH sensitivity. Then, by cross-liking NIPAAm, they could design and fabricated dual stimulus-responsive system to deliver berberine hydrochloride to the cancerous site. By changing pH and temperature NGs, networks were weakened, and the NGs collapsed to release drug rapidly. Also, the cytotoxicity test showed the low cytotoxicity and high biocompatibility [35]. Rao et al. fabricated poly(vinyl caprolactam) (PVCL) nanogels with disulfide linkages to deliver Dox for cancer treatment [36]. This system could release Dox under dual stimulus conditions, such as redox and temperature. As-mentioned nanogels were biocompatible against CCDK-skin fibroblast cells, and on the other hand, they showed high cytotoxicity against HepG2 cancer cells. Also, they could release Dox nearby nucleus by easy interrelation in the cancer cells [36]. Another pH and temperature-responsive Dox delivery system based on nanogels for cancer treatment is PNIPAAm and polyethylenemine (PEI) nanogel with magnetic graphene nanosheets as core of the system [37]. The LCST of this nanogel can be easily tuned in the range of 38–42°C. The biocompatibility and nontoxicity of the blank nanogel were confirmed against HEK293T normal and HepG2 cancerous cells and Dox loaded nanogels showed high cytotoxicity against HepG2 cell line with high cellular uptake [37].

In this research, a dual-responsive polymeric nanogel (P(VCL-co-AA)) was synthesized by free radical copolymerization of AA and VCL monomers. The synthesis process has been shown in Figure 1. Then, the P(VCL-co-AA), AA, VCL, Dox, and Dox-loaded nanogel were characterized by FT-IR. FE-SEM was used to visualize our nanogel before and after drug loading. DLS/Zeta potential technique was used to determine the particle size and distribution. Also, ^1^HNMR analysis was taken to structural characterization of nanogel. Dox loading efficiency, Dox controlled release, LCST, and swelling ratio of nanogel were studied to its drug delivery potential. Moreover, the biocompatibility of blank P(VCL-co-AA) against HFF-2 cell line and cytotoxicity of free Dox and Dox-loaded P(VCL-co-AA) against MCF-7 were studied by MTT assay.

## 2. Materials and Methods

### 2.1. Materials

Acrylic acid (AA) as a pH-responsive monomer, Vinylcaprolactam (VCL) as a temperature-responsive monomer, and triethylene glycol dimethacrylate (TEGDMA) were obtained from Merck Chemical Co. (Darmstadt, Germany). Potassium persulfate (KPS) was obtained from Sigma-Aldrich, Chemical Co. (St. Louis, MO USA). Sodium dodecyl sulfate (SDS) was obtained from Merck (Darmstadt, Germany). Doxorubicin (Dox) was obtained from Ebewe (Ebewe pharma, Austria). The cell culture medium (RPMI-1640), penicillin-streptomycin, and FBS were obtained from Gibco Company, Scotland. MCF-7 and HFF-2 cell lines were purchased from the Pasteur Institute, Iran. Dimethyl sulfoxide (DMSO), trypsin, and 5-diphenyl-2-H-tetrazolium bromide (MTT) were obtained from Sigma-Aldrich Chemical Co., USA.

### 2.2. Synthesis of Dual-Responsive Polymeric Nanogel

P(VCL-co-AA) nanogel was synthesized using TEGDMA as a cross-linker and KPS as a polymerization initiator. The P(VCL-co-AA) synthesis procedure was used. In a two-neck round bottom container, VCL (2.5 g), AA (0.075 ml), TEGMA (0.0774 g), KPS (0.425 g), and SDS (0.25 g) were dissolved in 30 ml water. Then, the mixture was purged under the nitrogen atmosphere and in an oil bath at 70°*C* for 24 h. After 24 h, we must cool it down to room temperature; then, we pass it from a filter paper then dry it in a freeze dryer.

### 2.3. Nanogel Characterization

Fourier transforms infrared (FT-IR) spectra of the P(VCL-co-AA), AA, VCL, Dox, Dox-loaded nanogel were taken in a Bruker tensor FT-IR (Bruker, Tensor 27, Germany). The samples were provided using potassium bromide (KBr) and then compressing the mixture to make disks. A scanning electron microscope (SEM) was used to visualize our nanogel and drug-loaded nanogel (MIRA 3 FEG-SEM, Tescan, Czech Republic). Proton nuclear magnetic resonance (1 222 H-NMR) spectra were documented at 25°C by an FT-NMR (400 MHz) Bruker spectrometer (Bruker, Ettlingen, Germany). The polymer for HNMR spectroscopy was provided by dissolving the P(VCL-co-AA) polymer in DMSO as a solvent. The average diameter and zeta potential of nanogel P(VCL-co-AA) and Dox-loaded nanogel were measured by laser-scattering technique (NanoZS ZEN 3600, Malvern Instruments, UK) before examination use of DMSO as a solvent.

### 2.4. Lower Critical Solution Temperature (LCST) Measurement

The LCST of nanogel was determined by the optical turbidity measurement method. A weighted amount of nanogel (0.1 g) was dissolved in buffers with various pHs (5, 7.4, 8) and the temperature was then gradually raised. The temperature at which detectable sediments were formed in the mixture was reported as nanogel LCST at relevant pH.

### 2.5. Swelling Ratio of P(VCL-co-AA) Measurement

For swelling ratio investigation, 0.3 g of dried nanogel was dissolved in 20 ml of water, then left for 72 hours to swell. The swelling ratio of P(VCL-co-AA) was calculated by following equation:

(1) $$\begin{array}{c} \text{Swelling ratio }\left(\%\right)=\frac{\text{Wt}–\text{Wd}}{\text{Wd}}*100. \end{array}$$

Wt is the swollen weight (gr), and Wd is the dried weight (gr).

### 2.6. Drug Loading into the Nanoparticles

Thirty milligrams of synthetized nanogel P(VCL-co-AA) was dispersed in 3 ml deionized water under stirring at 4°C. Then, 2.25 ml Dox solution (50 mg DOX in 25 ml deionized water) was added, and the system was stirred at 400 rpm for 24 h. After that, the drug-loaded polymer was centrifuged (6000 rpm, 10 min). Then, drug-loaded nanogel was dried in a freeze dryer. The loading percentage was determined by a spectrophotometric method (UV-Vis) at 482 nm.

### 2.7. *In Vitro* Controlled dox Release

Dox-loaded P(VCL-co-AA) was dispersed in 5 ml of PBS with different pHs (7.4 and 5.4). The vials were transmitted into a shaker incubator at temperatures about 37 and 40°C. At specified intervals, the contents of the vials were centrifuged, and the supernatant was removed and replaced with a refresh PBS. The released drug amount was determined by a UV-Vis spectrophotometer at 482 nm.

### 2.8. Cell Culture

Cell culture was performed according to the method previously described [23, 38]. Briefly, human foreskin fibroblast (HFF-2, normal cell) was chosen for the evaluation of biocompatibility and safety of blank P(VCL-co-AA) on normal cells. Cytotoxicity evaluation of Dox-loaded P(VCL-co-AA) was evaluated on human breast cancer cells (MCF-7). The cell lines were incubated in RPMI 1640 medium (10% (*v*/*v*) FBS and 100 U/ml penicillin) at 37°C in a 5% CO_2_ humidified atmosphere [22, 39].

### 2.9. The *In Vitro* Cytotoxicity Using MTT Assay

The cytotoxicity of P(VCL-co-AA) against HFF-2 and Dox-loaded P(VCL-co-AA) cytotoxicity against MCF-7 cells was assessed *in vitro*. The cells were seeded into MTT microplates (96-well) with a density of 10^4^ cells/well and incubated for 24, 48, and 72 h. The HFF-2 cells were treated with blank P(VCL-co-AA) with 0.8 to 400 mg ml^−1^ concentration range. MCF-7 cells were treated with Dox-loaded P(VCL-co-AA) with concentrations ranging from 0.039 to 50 mg ml^−1^. After the incubation time was elapsed, the contents of the wells were replaced with 20 *μ*l MTT solution (5 mg/ml in PBS). After 3 h, the purple formazan crystals were formed. The crystals were dissolved with 100 *μ*l DMSO. For cell viability detection, the absorbance of microplate content was assessed at 570 nm with an Elisa microplate reader. All experiments were repeated three times [39, 40].

## 3. Results and Discussion

### 3.1. Structural Characterization

In order to structure characterization of nanogel in comparison with free monomers and FTIR measurements of monomers, polymeric nanogels were obtained and are illustrated in Figures 2(a)–2(c). However, for displaying Dox existence in polymeric nanogel after drug loading, the FT-IR analysis of free Dox and Dox-loaded sample was obtained and is shown in Figures 2(d) and 2(e). There were significant differences between the prepared polymeric nanogels and the monomers. The characteristic peaks of AA related to C=O and C=C bonds were located at 1635 and 1600 cm^−1^. After the polymerization process, as illustrated in Figure 2(c), the C=O bond was visible at a wavelength of 1635 cm^−1^ again. While the peak of the carbon-carbon double bond was removed, which indicates the successful synthesis of nanogel. Also, the peak in the wavelength of 1735 cm^−1^ has ascribed to the stretching vibration of -COOH. The broad peak from 2800 to 3500 cm^−1^ in Figures 2(a) and 1(c) is related to O-H stretching of AA carboxylic acid functional group [41]. The vibration of C-H bond due to C=C-H corresponding to AA can be seen at wavelength 980 cm^−1^ as shown in Figure 2(a). After polymerization, this peak has been removed in the FT-IR pattern, and instead, a peak is formed at 1161 cm^−1^, which corresponds to the C-C band. As shown in Figures 1(c), O-H group vibration of acrylic acid units is revealed at wavelength 3030 cm^−1^, in which after polymerization this peak is removed [41–43]. At the same time, the absorption peak of the C-H bond of methylene groups after polymerization is visible at 2927 cm^−1^ in the nanogel pattern [43]. Figure 2(b) shows the FT-IR spectrum of the VCL monomer. The peak generated at wavelengths of 1625 cm^−1^ corresponds to C=C, and the peak generated at 1660 cm^−1^ corresponds to the carbonyl group (C=O), which are two characteristic peaks of the VCL monomer. The peaks generated in positions 2937 cm^−1^ and 2851 cm^−1^ belong to the aliphatic C-H stretching band. At wavelength 1440 cm^−1^, the peak corresponding to -CH_2_- is displayed. The characteristic peaks of the vinyl group (=CH and =CH_2_) are located at 3108 cm^−1^ and 996 cm^−1^. Also, the peak of the C-N band is located at 1487 cm^−1^ wavelength [44]. The peak created at 3274 cm^−1^ also corresponds to the N-H band. After polymerization, as shown in Figure 2(c), the peak at position 1630 cm^−1^ belongs to the carbonyl group. The peak of the carbon-carbon double bond is also removed after polymerization. This phenomenon indicates that the polymerization process continues with the opening of the carbon-carbon double bond. The aliphatic C-H stretching is visible at wavelengths 2927 cm^−1^ and 2859 cm^−1^ as long as they were visible in the monomer patterns. The CH_2_ peak is located at 1420 cm^−1^ wavelength. Also, after polymerization, the peaks of the vinyl group are removed, which indicates a successful polymerization process. The peak corresponding to the stretching vibration of C-N is located at 1452 cm^−1^, and the peak at position 3274 cm^−1^ corresponds to the N-H band, which becomes broader in the polymer state [32, 44, 45]. Figure 2(d) shows the FT-IR profile of doxorubicin, and Figure 2(e) shows the Dox-loaded P(VCL-co-AA). In Figure 2(d), the peak created at position 1731 cm^−1^ corresponds to the C=O group of Dox. As shown in Figure 2(e), the intensity of this peak increased after the drug was loaded with P(VCL-co-AA). Also, peaks between 1400 and 1500 cm^−1^ wavelengths correspond to the doxorubicin's aromatic ring, and peaks around 1100 cm^−1^ are also related to the C-O bond [46–48]. The doxorubicin aromatic ring peaks can also be seen in the drug-loaded nanogel. The above observations indicate the successful loading of doxorubicin into the nanogel.

The ^1^H NMR spectra of the P(VCL-co-AA) in DMSO are shown in Figure 3. The created peaks were named according to their molecular structure, as drawn in Figure 3. The protons in CH_2_ (peak a) of the carbon-carbon chain of copolymer were observed at 1.65 ppm. Peak b at 5.02 ppm is related to methylene resonance which bonded with N. The proton signals at 3.2 (peak c) and 2.6 ppm (peak d), respectively, have belonged to methine connected with N, and methylene bonded with a carbonyl group on the heterocyclic ring. Also, protons located in the heterocyclic ring were observed at 0.85 and 1.26 ppm (peak e). Protons in CH2 (peak f) of the carbon-carbon chain of nanogel were observed at 1.51 ppm. The peak observed at 2.3 ppm (peak g) have attributed to protons in the methine group of nanogel. According to meager amount of cross-linker in the reaction mixture, however, the characteristic peaks of TEGDMA appeared as weak peaks in the 1H NMR pattern which are located at 2.07 (peak h), 4.22 (peak i), and 3.7 ppm (peak j). Also, the signal at 7.4 ppm (peak k) can be related to protons, which are created by N hydrogen banding.

## 4. Physicochemical and Morphological Characterization

The size and surface charge of blank and Dox-loaded polymeric nanogels were assessed with DLS and zeta potential measurements, respectively. The size distribution of P(VCL-co-AA) and Dox @ P(VCL-co-AA) is illustrated in Figure 4. DLS demonstrated that the size of blank P(VCL-co-AA) is about 798 nm, but more than five times increases in the size of nanogel after Dox loading (4575 nm). Results of zeta potential measurement match the trend seen in DLS. Blank P(VCL-co-AA) and Dox-loaded P(VCL-co-AA) have a zeta potential of -30 and -20 mV, respectively. The pKa of Dox is about 8.46, which can be protonated under neutral conditions and be a positively charged molecule [49]. So, in the presence of Dox molecules in the P(VCL-co-AA) network, the surface charge decreases to -20 mV. In this state, the repulsive force between the Dox @ P(VCL-co-AA) nanoparticles reduces, and nanoparticles become aggregate with a larger size compared to blank P(VCL-co-AA).

The FE-SEM images of P(VCL-co-AA) and Dox @ P(VCL-co-AA) were taken for morphological property investigation, which illustrated in Figures 5(a) and 4(b), respectively. The dominant morphology of nanogels was spherical. Specifically, after Dox loading in nanogel, the aggregation of nanoparticles was slightly increased, and the empty spaces between nanoparticles reduced. As mentioned previously, after positively charging doxorubicin loading, the surface charge of P(VCL-co-AA) became lower. So, the repulsive force between the Dox-loaded nanogels has been reduced, and their agglomeration has been raised. The diameter of P(VCL-co-AA) was estimated 182.3 nm. In contrast, the estimated diameter of Dox @ P(VCL-co-AA) was about 115 nm. Evidence shows that the size of nanoparticles has decreased after doxorubicin loading. It can be due to pH-responsive behavior of P(VCL-co-AA) in the presence of Dox. P(VCL-co-AA) has become compact in the presence of the positively charged Dox, which has reduced its size after loading with the Dox. In summary, after Dox loading by P(VCL-co-AA), the diameter of the polymeric nanogels becomes smaller, and their aggregation increases. It is noteworthy that the hydrodynamic size calculated from DLS was larger than that observed by SEM, due to the highly swollen feature of P(VCL-co-AA) and Dox@P(VCL-co-AA) in an aqueous solution [50]. Moreover, they have significantly been shrunk under dry conditions [50]. The particle size distribution of P(VCL-co-AA) and Dox@P(VCL-co-AA) is illustrated in Figure 6.

### 4.1. LCST and Swelling Ratio of P(VCL-Co-AA)

Temperature-responsive polymers are transparent at temperatures below their LCST, but as the temperature rises, the polymer collapses and the solution become turbid. The LCST point of P(VCL-co-AA) was measured by assessing the phase transition of the nanogel solution in the distilled water at different pHs (5, 7.4, and 8). The results of LCST determination are reported in Table 1. As can be derived from the results, with decreasing pH, the LCST of the nanogel also augments, and this behavior indicates the sensitivity of the nanogel to the pH. Also, P(VCL-co-AA)'s swelling ratio was determined to be 160% after floating in the water at laboratory temperature after 72 hours. All evidence suggests that the synthetic copolymer is sensitive to temperature and acidity.

### 4.2. *In Vitro* Stimulus-Responsive Drug Release

Dox as a model chemotherapeutic drug was loaded in P(VCL-co-AA) nanogel. The Dox loading percentage was about 83% which was a significant amount.  Figure 7 presents the release of Dox-loaded in the P(VCL-co-AA) for 250 hours at temperatures of 37 and 40° C for pH 5.4 and 7.4. At first 12 h, Dox has bursting release. As shown in Figure 5, most drug release has occurred under 40°C (highest temperature) and pH 5.4, which has simulated conditions for drug delivery to the tumor. According to the release profile, the release rate at pH 7.4 and 37°C was higher than pH 5.4 and 37° C. This was due to using acrylic acid monomer as a pH-sensitive agent. Due to the presence of COOH groups in the structure of polyacrylic acid, when the pH is higher than acrylic acid's pKa (4.7), these groups are ionized and become to the COO^−^ form, which swells by repelling each other [22, 23]. During swelling, the synthesized nanogel particles separate, and the release of the drug occurs more efficiently and faster due to the gaps created in the nanocarrier's structure. However, with the increase of temperature to 40°C, a significant rising in drug release can be observed, especially in the pH of 5.4. This behavior is due to the change in phase of the VCL polymer and temperature-responsive feature.

### 4.3. *In Vitro* Cytotoxicity Using MTT Assay

The HFF-2 cell-line was chosen to investigate the blank P(VCL-co-AA) toxicity on normal cells by MTT assay. P(VCL-co-AA) polymeric nanogel was treated with the HFF-2 cell line and incubated for 24, 48, and 72 h. As illustrated in Figure 8(a), polymeric nanogel has no significant and detectable toxicity on HFF-2 cells even in the high P(VCL-co-AA) concentrations. In previous studies, the biocompatibility of polymers resulting from the polymerization of acrylic acid and vinyl caprolactam monomers was confirmed. The results of this study also confirmed the biocompatibility of TEGDMA cross-linker.  Figure 8(b) illustrates the cytotoxicity of drug-loaded P(VCL-co-AA) on the MCF-7 cell line at concentrations ranging from 0.039 to 50 *μ*g mL^−1^ for 48, 24, and 72 hours. By Dox concentration increment, the MCF-7 cells' viability decreased, and with increasing incubation time, the toxicity of Dox-loaded P(VCL-co-AA) augmented. So, Dox-loaded P(VCL-co-AA) at different incubation times has concentration-dependent toxic effects on MCF-7 cell line, which indicates the release of the drug from the designed drug delivery system under cancerous site condition. As can be seen in Figure 8(c), with free Dox concentration augment, the cell viability decreases, and with increasing incubation time, the toxicity of the drug on cells rises. For example, the vital activity of the cells at a concentration of 50 *μ*g ml^−1^ is 77.7% at 24 hours of incubation time, 74% at 48 hours of incubation time, and 25% at 72 hours of incubation time. Comparing Figures 8(b) and 7(c), it can be concluded that in all three time periods, the toxicity of the Dox-loaded P(VCL-co-AA) is higher than that of free Dox, which indicates the high efficiency of the synthesized nanogel. Enhanced toxicity of Dox-loaded P(VCL-co-AA) on MCF-7 cell line compared to the free Dox would be a massive benefit in reducing the drug dose and its side effects in the clinical cancer treatment applications.

## 5. Conclusion

The results this research have shown that the dual responsive cross-linked P(VCL-co-AA) nanogel can be synthesized through the free radical copolymerization-crosslinking method with a high yield. The copolymer obtained has a nanogel structure.

The characteristic properties of the nanogel were investigated by FT-IR, H-NMR, SEM, and DLS analysis, which confirmed the successful synthesis with suitable physicochemical properties. This system showed a significant loading of Dox (83%). Release in the simulated tumor area was higher than physiological conditions. The biocompatibility of nanogel was proved by MTT assay on HFF-2 cell line. The *in vitro* cytotoxicity evaluations of Dox-loaded P(VCL-co-AA) nanogel on MCF-7 cell line showed high cytotoxic effect compared to free drug. In general, these characteristics indicate the high efficiency of this specially designed smart drug delivery system for treatment of breast cancer.

### 5.1. Future Perspectives

The existence of some marketed formulation of nanogels shows the effective and successful performance of this class of nanocarriers in pharmaceuticals for preclinical and clinical applications. However, there are a number of inadequacies for their scale-up that future research should address. Development of a cost-effective and stable procedure for repeatable synthesis of nanogels is essential for their future marketable application. Therefore, despite the huge progress in creating stimulus-responsive nanogels for cancer treatment, still a lot of work is required to be done for their scaling up.

## Figures and Tables

**Figure 1:** Synthesis process of dual-responsive P(VCL-co-AA) nanogels.

**Figure 2:** FT-IR spectra of (a) AA, (b) VCL, (c) P(VCL-co-AA), (d) Dox, and (e) Dox @ P(VCL-co-AA).

**Figure 3:** ^1^H NMR spectra of the P(VCL-co-AA).

**Figure 4:** Size distribution analysis by dynamic light scattering (DLS).

**Figure 5:** SEM images of P(VCL-co-AA), (a) scale bar 500, and (b) 200 nm and Dox @ P(VCL-co-AA), (c) scale bar 500, and (d) 200 nm.

**Figure 6:** Particle size distribution of (a) P(VCL-co-AA) and (b) Dox-loaded P(VCL-co-AA).

**Figure 7:** DOX release profile at various pH and temperature.

**Figure 8:** The cytotoxicity of (a) blank P(VCL-co-AA) to HFF-2 clell line, (b) Dox @ P(VCL-co-AA), and (c) Dox to MCF-7 cell line.

**Table 1:** LCST points of P(VCL-co-AA) in various pHs.

pH	5	7	8
LCST (°C)	17-20	25-28	32-34

## Data Availability

All data used to support the findings of this study are included in the article.

## Abbreviation

AA: Acrylic acid
DLS: Dynamic light scattering
EE: Encapsulation Efficacy
FBS: Fetal Bovine Serum
FE-SEM: Field Emission Scanning Electron Microscopes
FT-IR: Fourier Transform-Infrared Spectroscopy
^1^HNMR: Hydrogen-Nuclear Magnetic Resonance
IC_50_: Inhibitory Concentration of 50%
LCST: Lower critical solution temperature
NIPAM: N-Isopropyl acryl amide
NG: Nanogel
VCL: Vinylcaprolactam
TEGDMA: Polyethylene glycol dimethacrylate
KPS: Potassium peroxydisulfate
SEM: Scanning Electron Microscopy
SDS: Sodium dodecyl sulfate
DMSO: Dimethyl sulfoxide.
